The article "Computer-Aided Design and Computer-Aided Manufacturing (CAD/CAM) Complete Dentures for Atrophic Alveolar Ridges: Workflow Combining Conventional and Novel Techniques" was published in 2022. Journal: Cureus.

# Computer-Aided Design and Computer-Aided Manufacturing (CAD/CAM) Complete Dentures for Atrophic Alveolar Ridges: Workflow Combining Conventional and Novel Techniques

**DOI:** 10.7759/cureus.21093

**Published:** 2022-01-10

**Authors:** Carlos Jurado, Mohammed Sayed, Chin-Chuan Fu, Jose Villalobos-Tinoco, Akimasa Tsujimoto

**Affiliations:** 1 Prosthodontics, Texas Tech University Health Sciences Center El Paso Woody L. Hunt School of Dental Medicine, El Paso, USA; 2 Prosthetic Dental Sciences, Jazan University College of Dentistry, Jazan, SAU; 3 Restorative Dentistry, University of Alabama at Birmingham School of Dentistry, Birmingham, USA; 4 Oral Rehabilitation, Autonomous University of Queretaro School of Dentistry, Queretaro, MEX; 5 Operative Dentistry, The University of Iowa College of Dentistry and Dental Clinics, Iowa City, USA

**Keywords:** alveolar ridge, digital dentistry, complete denture prosthesis, cad/cam, dentistry

## Abstract

Extreme residual ridge resorption is a challenging clinical situation for the fabrication of complete dental prostheses. Computer-aided design and computer-aided manufacturing (CAD/CAM) complete dentures have been shown to have superior fit and material strength to conventionally fabricated dentures, but no clinical protocols have been described for cases of extreme residual ridge resorption. This report describes a workflow combining conventional and novel techniques for CAD/CAM complete dentures fabrication for atrophic alveolar ridges and demonstrates that a CAD/CAM workflow is an effective tool for solving this complex situation.

## Introduction

It has been shown that edentulism is the final result of a multifactorial process comprising biological and patient-related factors [1]. Complete edentulism has decreased in developed countries, but it still remains a significant problem a group that varies from 15% to 54% of the senior population [2]. Removable complete dentures are the least invasive and most affordable option for the prosthodontic rehabilitation of edentulous patients [3]. Treatment of edentulous patients with full complete dentures demands many technical steps, in which making accurate impressions is considered to be essential [4]. Well-fitted removable complete dentures reduce the occurrence of traumatic ulcers and show higher comfort when wearing prostheses [5]. Denture retention is vital for masticatory function and speech, and can provide a good quality of life [6]. The traditional techniques for denture fabrication require a high level of knowledge and skillful manipulation of the materials, which may lead to multiple errors during denture fabrication [7]. Moreover, the production of complete dentures using conventional techniques and materials such as monomers can cause an allergic reaction in some patients, regardless of the curing method [8]. Fortunately, all of these problems have been solved by the digital workflow for denture fabrication, because milled resin pucks contain negligible unpolymerized monomers, the dentures are made from highly crosslinked pucks, and fabrication time is considerably decreased, even if novel and traditional fabrication are combined [9]. Furthermore, recent studies have claimed higher retention and fit of computer-aided design and computer-aided manufacturing (CAD/CAM) fabricated dentures than those conventionally fabricated [10].

CAD/CAM dentures can be fabricated within hours, whereas conventional techniques can require days for production [11]. Therefore, the development of novel technologies in dentistry is allowing clinicians to make restorations in a faster, easier, and more accurate manner. New techniques in dentistry have countless applications, such as onlay, crown, and bridge, and the production of a completely removable prosthesis is one of them [12]. These novel techniques allow the clinician the option to fabricate complete dentures in the office, in a laboratory, or at a centralized production center [13]. The practice of making complete removable dentures using subtractive technology has become very common and continues to spread, and the literature provides reports describing both fully digital and combinations of digital and conventional methods for their production [14]. However, no clinical reports have described complex clinical situations with patients presenting atrophic alveolar ridges. Therefore, this article aims to report a method combining novel and traditional methods for the fabrication of CAD/CAM complete dentures for a patient presenting with atrophic alveolar ridges. Moreover, this workflow could be used for clinicians with no access to CAD/CAM technology in their offices.

## Technical report

A female patient, 45 years of age presented to the clinic with the chief complaint of needing new dentures. The patient claimed to have been wearing the existing complete dentures for the past 15 years (Figures 1-3).

**Figure 1:** Initial complete dentures for intra-oral frontal view

**Figure 2:** Initial complete dentures for intra-oral frontal view

**Figure 3:** Initial smile

After a detailed evaluation, the findings were extreme alveolar ridge resorption in the maxilla and mandibular arches, and the case was diagnosed as a Class III complete edentulism. The alveolar mucosa appears healthy with adequate keratinized gingiva covering the crest of both ridges, although it seems thinner relative to the mandibular arch (Figures 4-6).

**Figure 4:** Initial intra-oral without dentures for maxilla view

**Figure 5:** Initial intra-oral without dentures for mandible view

**Figure 6:** Initial intra-oral without dentures for intra-oral frontal view

The patient reported the extraction of all her teeth for various reasons, such as caries and periodontal disease in young adulthood. The teeth of complete denture showed severe wear, which caused a non-ideal smile line. Due to the known pattern of maxillary and mandibular ridges resorption and the loss of the vertical dimension of occlusion resulting from wear of the denture teeth, the denture occlusion became Class III.

Treatment options were explained to the patient; however, treatment had to start with a new set of complete dentures, before the work necessary for a fixed mandibular implant-supported prosthesis could be done. The patient accepted and she was offered the option to have milled complete dentures. However, due to the extreme alveolar ridge resorption, it was suggested that the final impressions, master cast fabrication, and jaw relation records should be completed using conventional techniques. The patient accepted the proposal and requested the start of treatment. 

The maxillary and mandibular complete denture bases presented good retention and because of the severe bone atrophy, it was decided to use the current prostheses as custom impression trays. Conventional border molding with green compound (Kerr Impression Compound sticks, Kerr Corporation, Orange, California, USA) was used to record the tissues in functional form. The areas were recorded by manipulating the tissues through outward, inward, forward and backward movement. Final impressions with polyvinyl siloxane (PVS) material (Aquasil® Ultra+ Smart Wetting Impression Material, Dentsply Sirona, Charlotte, North Carolina, USA) were made using her current prostheses, and they were poured out and master casts were fabricated with type IV stone (ResinRock, Whip Mix Corporation, Louisville, Kentucky, USA). Conventional jaw relation records using record bases (Triad® VLC Denture Base Material, Dentsply Sirona) with pink u-shaped occlusal rim wax (HYGENIC® Wax, Coltene Whaledent, Inc, Cuyahoga Falls, Ohio, USA) and vinyl polysiloxane bite registration (Regisil® Rigid Digit®, Dentsply Sirona) were fabricated following traditional record measurements of closest speaking space, lip support, and smile line in order to obtain the vertical and vinyl polysiloxane bite registration (Figure 7). 

**Figure 7:** Conventional maxillomandibular relationship

A laboratory order form was downloaded from the company’s website and filled out. The clinician and patient selected the tooth shape, tooth shade, denture base shade, and anatomic features to be included in the denture base. Mounted casts, jaw relations records, and complete laboratory prescription forms were shipped to the company (AvaDent® Digital Dental Solutions, Scottsdale, Arizona, USA). A few days later the company provided a password to the clinician in order to log in to the company’s website where the tooth arrangement and all other features requested were digitally designed. The clinician was able to digitally modify the tooth arrangement for every individual tooth if desired, and the system also provided the option to alter the anatomic features requested in the prostheses (Figures 8-9).

**Figure 8:** Digital denture designing for digital teeth positioning

**Figure 9:** Digital denture designing for digital teeth selection

The company mailed the prostheses the following week, and the patient was scheduled for a delivery appointment (Figures 10-11). 

**Figure 10:** Milled CAD/CAM complete dentures (frontal view) CAD: Computer-Aided Design; CAM: Computer-Aided Manufacturing

**Figure 11:** Milled CAD/CAM complete dentures (lateral view) CAD: Computer-Aided Design; CAM: Computer-Aided Manufacturing

The milled complete denture prostheses were tried in, and they provided acceptable retention and stability. White pressure-indicating paste (Mizzy Pressure Indicating Paste (PIP), Mizzy Inc., Cherry Hill, New Jersey, USA) was used in order to evaluate the fit and pressure areas in the intaglio surfaces of the prostheses and no adjustments were needed. Border extensions were also assessed using disclosing wax (Disclosing Wax™, Kerr Corporation). A conventional clinical remount was made in order to evaluate occlusion. No occlusal adjustments were required. Phonetics and esthetics were evaluated and both patient and clinician were satisfied (Figures 12-14). 

**Figure 12:** Placement CAD/CAM complete dentures for intra-oral frontal view CAD: Computer-Aided Design; CAM: Computer-Aided Manufacturing

**Figure 13:** Placement CAD/CAM complete dentures for intra-oral lateral view CAD: Computer-Aided Design; CAM: Computer-Aided Manufacturing

**Figure 14:** Postoperative smile

The manufacturing software allows full control over the selection of denture tooth position, shape, cuspal inclination, and occlusal relationship upon centric and eccentric movements. Since the patient presented with an atrophic mandibular ridge, semi-anatomic acrylic resin teeth of 15 degrees were chosen for the posterior teeth, which were set over the crest of the ridge in a bilateral balanced occlusal scheme to allow maximum denture stabilization upon horizontal jaw movements. The patient was seen in a follow-up appointment on the next day and no complaint regarding the prostheses was noted. The patient was satisfied with the prostheses’ retention, stability, and aesthetics. The clinician evaluated the denture foundation areas and no sore spots were present; pressure-indicating paste was used again in order to assess the fit and pressure areas in the intaglio surfaces of the prostheses and no denture adjustment was required. The one-week and two-week follow-up appointments showed complete patient satisfaction with no need for denture adjustment following thorough intra-oral evaluation.

## Discussion

Extreme residual ridge resorption is a challenging clinical situation for the fabrication of complete dental prostheses and there are no published technical reports of CAD/CAM workflows for a complete prosthesis solving this complicated situation. This workflow combines traditional and novel techniques in order to fabricate digital complete dentures in a patient presenting extreme alveolar ridge atrophy. Due to the short height of the ridge, it was decided to take a conventional final impression following the functional impression technique, using her current complete dentures. Making the final impression using the patient’s existing denture as the impression tray has been shown to be a successful approach for atrophic ridges. Conventionally mounted master casts can either be scanned by the clinician or simply mailed to a dental laboratory. Once the digital file has been created, the computerized designs for the complete removable dentures are made, and the clinician can access them online with full control of the tooth shape, shade and arrangement, denture plate color, and anatomical features. After the dentist approves all the features, the company ships the restorations with little delay.

This technique is not fully digital fabrication, and there is a need for combining conventional techniques and digital dentistry workflow. Clinicians need to make a good traditional PVS impression covering all the landmarks needed for complete dentures and this may be technique sensitive. The combined technique here using the conventional and novel technique is unique, no dental laboratory companies have described it. A few companies only offer fully digital techniques; however, those techniques are recommended for patients with good bone levels, not atrophic maxilla and mandible like in our presented case.

Wearing a complete denture for several years may have adverse effects on the alveolar ridge bone as well as on the keratinized mucosa, and wearing unstable dentures may cause adverse effects such as extreme atrophy of the alveolar ridge [15]. Mandibular ridge atrophy is sometimes so advanced that the low mandibular height. makes it almost impossible to deliver stable and well-functioning complete dentures with conventional techniques, which leads to chewing difficulties, pain, sore spots, and poor oral health, which in turn impair quality of life. Unfortunately, due to the high costs of implant therapy, complete dentures are still the first choice of treatment for patients with financial constraints, so it is imperative to supply a well-fitting prosthesis in order to improve the patients’ quality of life.

Milled complete dentures can be either fabricated all in one piece with the base plate and teeth together or separated, as in this case report, where the denture base is milled from one puck and the teeth from another. Milling the two pieces separately provides higher aesthetic results because there are multi-chromatic discs offering shade gradation, which mill to give teeth with high aesthetics. Moreover, if a patient should break the teeth, it would be possible merely to mill the teeth and bond them to the existing plate, without the need to mill an entirely new base plate.

There are numerous techniques for making final impressions with edentulous arches [16]. This clinical situation was complex because the patient had been wearing the existing complete dentures for the last 15 years and the residual alveolar ridges in the mandible were excessively reabsorbed and atrophied. Due to the low height of the ridge, it was decided to make a conventional final impression following the functional impression technique using her current complete dentures. Making the final impression using the patient’s existing denture as the impression tray has been shown to be a successful approach for atrophic ridge [17]. Unfortunately, the patient needs to wait in the dental clinic while the clinician pours the impression and fabricates the conventional master cast.

Milled complete dentures, including the teeth, are made out of pre-polymerized resin acrylic pucks and teeth are bonded to the plate using a proprietary bonding mechanism in the milled recesses. This resin puck is produced under higher pressure and heat, thus polymerization shrinkage does not happen and porosity is reduced. The adherence of *Candida albicans* to the base plate also decreases [18] The absence of polymerization shrinkage in the complete milled dentures results in a highly accurate denture fitting and improvement of retention [19]. The CAD/CAM company provides the clinician with the opportunity to select the shade of the denture teeth, anatomic features of the denture base, and modifications to the teeth set-up before milling the final prosthesis.

Incorporating new technology or clinical techniques can be challenging because clinicians need to become familiar with the software and operating equipment used by the dental laboratories to maximize the options for patient care. Due to the investment in novel equipment, laboratory costs may be increased compared with conventional methods. A previous study comparing the trueness fit of the intaglio surface of conventional and CAD/CAM dentures demonstrated that the conventional prosthesis is better [20]. However, as technology improves, the present case report successfully combines the advantage of CAD/CAM technology and traditional clinical recording methods for the construction of complete dentures in atrophic alveolar ridges. The presented workflow is completely functional because the clinician does not need to have either an intraoral or laboratory scanner to offer CAD/CAM dentures to patients. Following this protocol, the clinician can do conventional final impressions, jaw relation records, and mounting, then send those records to the laboratory in order to fabricate CAD/CAM dentures. If the dental office has a laboratory scanner, the records could be scanned and the stereolithography (STL) file sent to the company. This combined workflow offers critical information about the maxillomandibular relationship provided by conventional techniques and the improved material properties and fit of milled dentures.

## Conclusions

Combining traditional and novel technology for CAD/CAM complete dentures can provide clinically acceptable results for complex clinical situations such as extreme alveolar ridge atrophy. Conventional impression techniques for the impression of the denture foundation areas can accurately capture all features and novel CAD/CAM manufacture offers improved denture materials and enhanced fit, retention, and stability of the prostheses. The presented clinical protocol may be followed in compromised clinical situations to achieve clinically acceptable results.
